# Expression-EEG Bimodal Fusion Emotion Recognition Method Based on Deep Learning

**DOI:** 10.1155/2021/9940148

**Published:** 2021-05-25

**Authors:** Yu Lu, Hua Zhang, Lei Shi, Fei Yang, Jing Li

**Affiliations:** ^1^Fuyang Vocational and Technical College, Fuyang, Anhui 236031, China; ^2^Department of Electrical & Information Engineering, Sichuan Engineering Technical College, Deyang, Sichuan 618000, China

## Abstract

As one of the key issues in the field of emotional computing, emotion recognition has rich application scenarios and important research value. However, the single biometric recognition in the actual scene has the problem of low accuracy of emotion recognition classification due to its own limitations. In response to this problem, this paper combines deep neural networks to propose a deep learning-based expression-EEG bimodal fusion emotion recognition method. This method is based on the improved VGG-FACE network model to realize the rapid extraction of facial expression features and shorten the training time of the network model. The wavelet soft threshold algorithm is used to remove artifacts from EEG signals to extract high-quality EEG signal features. Then, based on the long- and short-term memory network models and the decision fusion method, the model is built and trained using the signal feature data extracted under the expression-EEG bimodality to realize the final bimodal fusion emotion classification and identification research. Finally, the proposed method is verified based on the MAHNOB-HCI data set. Experimental results show that the proposed model can achieve a high recognition accuracy of 0.89, which can increase the accuracy of 8.51% compared with the traditional LSTM model. In terms of the running time of the identification method, the proposed method can effectively be shortened by about 20 s compared with the traditional method.

## 1. Introduction

Emotional computing is widely used in the fields of games, mental health, learning, and education. The goal is to develop a computing system that can carry out “emotional communication.” It is required that the algorithm's type recognition, degree judgment, and feedback speed of emotions should be as close as possible to real human emotional responses [1–4]. As one of the key issues in the field of emotional computing, emotion recognition has rich application scenarios and important research value and has attracted widespread attention in recent years [5–7]. Taking medical work as an example, real-time and accurate grasp of the physical and psychological conditions of unconscious patients play an important role in the recovery of patients. Therefore, it is of great significance to use the existing pattern recognition technology to study difficult problems such as the physical condition of unconscious patients.

Emotion recognition methods can be divided into two categories: single-modality and multimodality [8–10]. Single-modal data acquisition is easier, and analysis methods are more mature. Therefore, most previous researches focused on monomodal emotion recognition, that is, emotion recognition for a pattern of data, such as traditional audio, facial expressions, physiological signals, or a certain form of data in text and body movements [11].

Multimodal emotion recognition can use all the characteristics of different signals such as human expressions and brain signals, so that the complementary characteristics of multiple modalities in expressing emotions are reflected in the final algorithm results, thereby improving the recognition accuracy [12, 13].

As the product of current artificial intelligence technology and big data collection, deep neural network combines multimodal emotion recognition methods with deep learning networks. Through multilayer network model iterative training and learning [14, 15], the signal data can be extracted and calculated effectively. And based on the continuous learning of its own network, the network model parameters can also be adjusted in time. The problem of feature redundancy and lack of key features is solved, and the corresponding emotion recognition performance is improved.

The rest of this article is organized as follows. The second chapter introduces the related research in recent years. The third chapter introduces the bimodal emotion recognition method based on deep learning, including facial expression feature extraction and EEG signal features. The fourth chapter introduces the experimental simulation analysis of the feasibility and optimality of the method proposed in this paper based on the MAHNOB-HCI data set. The fifth chapter is the conclusion of this article.

## 2. Related Works

In recent years, researchers have conducted extensive research on various types of modal information that can express emotions. Studies have found that changes in human emotions can cause changes in expression, behavior, psychology, and physiology. Among them, facial expressions, postures, and physiological signals can independently express certain emotions [16–18].

In the research of monomodal emotion recognition, video, speech, text, and physiological signals all have certain expressions of emotion. Reference [19] uses ConvNet and DBNs to obtain information from videos, which has good performance on some emotions. Reference [20] summarized the methods and achievements of emotion recognition using electroencephalogram (EEG) in recent years. Reference [21] uses the convolutional-recurrent neural network (CRNN) to perform emotion recognition on multichannel EEG data and achieves ideal results.

But it needs to be pointed out that these types of emotional information are comprehensively displayed in the process of people communicating with each other. At present, researchers found that unimodal data has certain restrictions on the expression of emotions, and each mode has different sensitivities to different emotions [22]. Since each modal has a certain expression of emotion, some researchers have begun to conduct multimodal fusion emotion recognition research. Reference [23] uses a dual-mode autoencoder to study the emotional performance of EEG and eye movement signals. Experiments show that compared with the fusion of the two, the effect of identifying EEG features and eye movement features separately is poor. Reference [24] introduced a new method of modeling spatiotemporal information using three-dimensional convolutional neural networks (C3D) and combined it with a multimode deep belief network (MMDBN), which can represent audio and video stream cascades. Experiments on the eNTERFACE multimodal emotion database show that this method improves the performance of multimodal emotion recognition and is significantly better than the latest research scheme. Reference [25], based on the radial basis function and support vector machine network model, proposed a multimodal emotion recognition metric learning (MERML); a unified analysis of audio and video has a good performance in emotion recognition. This type of method usually only combines features by simple splicing, which easily causes feature redundancy. For video signals containing very large sample data, this will cause unnecessary experimental costs.

At the specific algorithm level of multimodal emotion recognition, with the breakthrough of deep learning methods in the computer field, neural network models are gradually applied to emotion recognition tasks [26]. The recurrent neural network (RNN) model has received extensive research and attention due to its obvious advantages in processing sequence tasks. Although recurrent neural networks can rely on cyclic connections to capture certain sequence context information, RNNs have the problem of vanishing gradients during back propagation. That is, as the number of neural network layers increases, the amount of values transferred is small and cannot cause parameter disturbances. An effective technology to overcome the problem of RNN gradient disappearance is adopted, namely, the Long Short-Term Memory (LSTM) network [27]. The LSTM network structure selectively “forgets” some inputs and “shields” some outputs through the “gate” structure so as not to affect the weight update of the next layer, so that the LSTM network can learn the best timing information related to the classification task [28]. In emotion recognition tasks, because of the continuity of facial expressions and EEG signals, emotional expressions are highly correlated in time series. However, single-point facial expression pictures and EEG signal data are often in the process of facial expression changes, which are prone to misjudgment [29, 30]. Therefore, for sequence emotion recognition tasks, LSTM's processing of sequences is similar to the processing method of the human brain on emotion recognition tasks, and the algorithm has the advantage of natural adaptability.

In view of the existing research work on emotion recognition, this paper proposes a deep learning-based expression-EEG bimodal fusion emotion recognition method. The main contributions are as follows:

1. Aiming at the problem of low accuracy of single-modal emotion recognition, combined with the advantages of human expression signal recognition and EEG signal emotion recognition, the accuracy of emotion recognition is improved, and the six emotions of anger, disgust, fear, happiness, sadness, and surprise are realized via accurate classification and identification
2. Facing the recognition accuracy and real-time requirements of emotion recognition models, it is based on the improved VGG-FACE network to realize the extraction of expression features and EEG features. First, the self-attention mechanism is introduced between the hierarchical networks to better distinguish each training layer and enhance the robustness of the system. The penalty term is introduced in the loss function to further improve the network and realize the diversification of the state vector of each layer. At the same time, it reduces the time of model training and learning and has a good recognition effect

## 3. Bimodal Emotion Recognition Method Based on Deep Learning

### 3.1. Expression-EEG Interactive Emotion Recognition Model

The system framework is shown in Figure 1. The LSTM emotion recognition model proposed in this paper for interactive collaboration between EEG signals and face video mainly includes two stages: feature extraction and interaction collaboration. In the feature extraction stage, first select key signal frames that need to be focused for data preprocessing and then extract features with strong expression and generalization capabilities. In the interactive collaboration stage, the features of the two modalities are first fused and learned. The special feature is that this article will also use the spatial frequency band attention mechanism to calculate the importance of the visual images of the *α*, *β*, and *γ* waves in the EEG signal. Reinforcement learning (RL) is performed through the time-domain attention mechanism to calculate the key signal frame time information that needs to be focused at the next time point and feed it back to the feature extraction stage. Finally, the emotion recognition result is outputted by the emotion classifier. Under this model, a closed loop is formed between the input signal and the model action—a process of selectively and repeatedly focusing on the multimodal signals of human emotions for emotion recognition.

### 3.2. Facial Expression Extraction

This paper uses fine-tuning to complete the retraining of the pretrained network. The advantage of fine-tuning is that you can use limited data to make the model achieve the desired effect. This paper uses the face data set FER2013 (the Facial Expression Recognition 2013 Dataset) to fine-tune the existing VGG-FACE network.

VGG-FACE is a 16-layer or 19-layer CNN architecture developed by the Visual Geometry Group (VGG) of Oxford University, which performs well in face recognition tasks [31]. Unlike VGG trained on the ImageNet data set, VGG-FACE is trained on a data set that only contains face data. And a deep convolution neural network model (DCNN) without pretraining as a baseline for experimental comparison was also introduced.

All the above network models are fine-tuned using the FER2013 data set. It was verified on the FER2013 test set and SFEW validation set to observe its performance. The experimental results are shown in Table 1.

As can be seen from the data in the above table, most of the pretrained network experimental results are better than the DCNN without pretraining, because the pretrained network has better initialization model parameters. Whether it is on FER2013 or SFEW, the best results are the VGG-FACE network pretrained on the face data set. The network reached an accuracy of 89.21% on the FER2013 test set and an accuracy rate of 78.24% on the SFEW test set. According to the experimental results, this paper finally uses a pretrained 16-layer VGG-FACE network. The network is fine-tuned on FER2013, and the acquired features are outputted to the LSTM unit to identify timing features.

The attention mechanism can be introduced between the input and output of the model, so that the performance of the model can be improved [32]. As shown in Figure 2, the main working principle of the attention mechanism is as follows: imagine the elements in the source as a series of <*K*, *V*> data pairs, determine the element *Q*, calculate the correlation between *Q* and each *K*, obtain the weight coefficient of each *K* corresponding to *V*, and then perform weighting on *V* and get the final attention value *Y*_att_:

(1) $$\begin{array}{c} Y_{\text{att}}=\overset{l}{\underset{i=1}{\sum }}\text{S}\text{imilarity}\left(Q,K_{i}\right)\cdot V_{i}, \end{array}$$

where *l* represents the length of source, and the meaning of the formula is as described above. The self-attention mechanism does not refer to the attention mechanism between the target and the source but occurs between the internal elements of the source or target. The attention mechanism can be understood as the situation of *K* = *V* = *Q*. The self-attention mechanism can more easily capture the long-distance interdependent features in the input sequence.

In the applied stacked LSTM network, three LSTM stacks are used to ensure that the model can learn higher-level temporal feature representation. Sequence data operations based on LSTM mean that the addition of layers increases the abstraction level of the input observation time and has better expressive capabilities.

In order to make each layer of LSTM in the stacked LSTM network have different proportions, the network model in this paper is further improved, and a self-attention mechanism is introduced between each layer of the LSTM network. It is worth noting that, unlike the attention mechanism, it can be updated iteratively through its own information. The flowchart of this part of the method is shown in Figure 3. This network model is mainly composed of a stacked LSTM network embedded with a self-attention mechanism. The hidden state and unit state of the stacked LSTM are used as the input of the self-attention mechanism module, and the output is the corresponding weight vector.

(2) $$\begin{array}{c} u^{t}=v^{T}\tanh\left(W_{s}X_{t}+b\right), \end{array}$$

(3) $$\begin{array}{c} a^{t}=\text{Softmax}\left(u^{t}\right), \end{array}$$

where the dimension of vector **X**_*t*_ is *n* × *r*, the dimension of vector **W**_*s*_ is *r* × *d*_*a*_, **b** and **v**^*T*^ are vectors of dimension *d*_*a*_. **W**_*s*_, **b**, **v**^*T*^ are the parameters of the network model, and **X**_*t*_ is the input of the self-attention mechanism module, which represents the hidden state **Y**_*t*_ or the unit state **Z**_*t*_ of a certain layer in the stacked LSTM.

(4) $$\begin{array}{c} Y_{t}=\left(y_{t}^{\left(1\right)},y_{t}^{\left(2\right)},\cdots ,y_{t}^{\left(l\right)}\right), \end{array}$$

(5) $$\begin{array}{c} Z_{t}=\left(z_{t}^{\left(1\right)},z_{t}^{\left(2\right)},\cdots ,z_{t}^{\left(l\right)}\right). \end{array}$$

Dot multiplying the weight vector **a**^*t*^ with the state value of LSTM, we can get

(6) $$\begin{array}{c} G_{t}=a^{t}X_{t}, \end{array}$$

where **G**_*t*_ is the weighted vector **Y**_*t*_′ or **Z**_*t*_′ obtained after the stack LSTM is updated. After calculation by the self-attention mechanism, different weights can be assigned to each layer of the network in the stack LSTM according to their importance. The network has been optimized to a certain extent, and the expression ability of the hierarchical features is improved.

Since the self-attention mechanism between adjacent time steps tends to assign similar weights, this paper adds a penalty term to prevent this problem from occurring and makes the weight vectors of different levels more diverse. While optimizing the weight, the penalty term not only reduces the redundant feature information but also makes the hierarchical relationship in the stacked LSTM more differentiated. This paper uses the statistical variance method to optimize the network.

(7) $$\begin{array}{c} P=\frac{1}{T}\overset{T}{\underset{t}{\sum }}\overset{L}{\underset{i}{\sum }}\left({\left(\alpha_{ti}-\mu \right)}^{2}+{\left(\beta_{ti}-\eta \right)}^{2}\right), \end{array}$$

(8) $$\begin{array}{c} \mu =\frac{1}{L}\overset{L}{\underset{i}{\sum }}\alpha_{ti},\eta =\frac{1}{L}\overset{L}{\underset{i}{\sum }}\beta_{ti}. \end{array}$$

In the formula, *α*_*ti*_ and *β*_*ti*_, respectively, represent the attention weight of the hidden state and the unit state at different time steps and levels: minimize it together with the original loss function.

(9) $$\begin{array}{c} L_{d}=-\log\left(p\left(y\left|a\right.\right)\right)-P, \end{array}$$

where −log(*p*(*y*|*a*)) represents the cross-entropy loss function, *a* represents the actual output of the model, and *y* represents the sample label.

### 3.3. EEG Feature Extraction

#### 3.3.1. EEG Feature Collection

EEG signals are the distribution of potentials on the scalp produced by brain neuron activity and are usually obtained by using an EEG device. The electrodes placed on the scalp transmit the electrical signals generated by the brain to the signal collector and then perform preamplification and electronic filtering (such as a 50 Hz notch filter). Then, through the power amplifier and A/D converter, the analog signal is converted into a digital signal that can be processed by the computer and then transmitted to the computer for relevant analysis and processing.

According to the recommendations of the International Electroencephalography Society, the current electrode placement for EEG acquisition generally adopts the international 10/20 system standard, as shown in Figure 4. Divide the connecting lines of the root of the nasion, vertex, and inion in equal proportions of 10%, and then divide the connecting lines of the nasion, external, ear hole, and inion into 10 equal parts. The electrode position is determined according to the intersection of the concentric circle centered on the vertex and the radius, and most of them are placed at the position of an integer multiple of 10% or 20% of the connecting line, so it is called a 10/20 system. There are a total of 21 electrodes, of which A1 and A2 are reference electrodes, as shown in Figure 4(b). The beginning of each electrode name uses one or two letters to indicate its area, as shown in Table 2. After the electrode name, a number or letter is used to indicate the distance from the center. An odd number means the left brain, and an even number means the right brain: the larger the number, the farther away from the center line. The position of the center line uses the mark “z” to represent the number 0 to distinguish it from the letter O. Modern 32-lead or 64-lead electrode caps are also based on the 10/20 system expansion. However, it should be noted that different EEG systems often have different names for similarly located electrodes.

#### 3.3.2. Data Preprocessing

The EEG signal will be affected by the experimental equipment and the breathing movement of the collected person during the collection process. Noise may interfere with the EEG signal, making the measurement result of the original signal unreliable. The purpose of preprocessing is to improve the overall recognition quality of EEG signals for more accurate analysis and measurement. The main categories of noise are low frequency baseband drift (BW) caused by breathing and body movement, high frequency random noise caused by power system interference (50 or 60 Hz), muscle movement, and random offset caused by poor electrode contact with the muscle interference.

Figure 5(a) shows the original EEG signals collected. In the filtering process, a 35 Hz Butterworth filter and a 50 Hz power interference removal filter are designed to eliminate power frequency interference, myoelectric interference, and electromagnetic interference in most power systems. Then, the signal is filtered by wavelet packet decomposition to remove baseband drift, and the EEG signal that removes interference and baseband drift is shown in Figure 5(b).

#### 3.3.3. Feature Extraction Process

Face video is the facial activity signal of experimental participants collected by an ordinary camera, which belongs to the visual signal. The method of collecting EEG signals is to allow experiment participants to wear electrode EEG caps while watching emotion-inducing videos, so as to obtain EEG signals from 32 different positions on the human cerebral cortex. It is difficult to directly merge two heterogeneous signals. For this reason, this paper proposes to extract features with strong expression ability and generalization ability and at the same time make the features of the two modalities effectively interact and cooperate. For face videos, facial expression features are extracted based on VGG-FACE. The feature extraction process of the face video is as follows: first, the face area in the video frame is detected by the VGG-FACE model. Then, use the VGG-FACE model to extract features from the face area. Finally, use the fully connected layer to process the features and output the final feature vector **x**_*v*,*n*_.

The feature extraction of the EEG signal is more complicated: Firstly, the original EEG signal is removed by the wavelet soft threshold algorithm to remove artifacts, thereby obtaining a relatively pure signal. Then, the EEG signal is divided into segments with a duration of *T*. Next, extract the spectral energy information of the three brainwave frequency bands of *α* wave, *β* wave, and *γ* wave from the *t*^th^ segment data and visualize it on the 32 electrodes of the corresponding electrode caps to obtain the three frequency bands of EEG images. The rising *β* wave of human emotion activation will be significantly enhanced in the forehead. Finally, CNN is used to extract the layer features *e*_*α*,*n*_, *e*_*β*,*n*_, and *e*_*θ*,*n*_ of the EEG images of the three frequency bands to fuse, as shown in equations (10) and (11).

In the calculation, the spatial frequency band attention mechanism is used to calculate the importance *e*_*n*_′ of the three groups of features, and finally, the fully connected layer is used to process the *e*_*n*_′ output feature vector *x*_*e*,*n*_.

(10) $$\begin{array}{c} e_{n}^{\prime }=e_{\alpha ,n}\theta_{en,1}+e_{\beta ,n}\theta_{en,2}+e_{\theta ,n}\theta_{en,3}. \end{array}$$

In the formula, *θ*_*en*,1_, *θ*_*en*,2_, and *θ*_*en*,3_ represent the importance assigned to *e*_*α*,*n*_, *e*_*β*,*n*_, and *e*_*θ*,*n*_respectively:

(11) $$\begin{array}{c} \theta_{en,i}=\frac{\exp\left(W_{h,i}h_{n-1}+b_{n,i}\right)}{\sum_{j=1}^{3}\exp\left(W_{h,j}h_{n-1}+b_{n,j}\right)},i=1,2,3. \end{array}$$

In the formula, *W*_*h*,*i*_ represents the weight matrix to be learned, *b*_*n*,*i*_ represents the deviation, and *h*_*n*−1_ represents the hidden state of the multilayer LSTM at a time point *n* − 1.

### 3.4. Expression-EEG Bimodal Fusion Emotion Recognition

This paper integrates facial expressions and speech signals for emotion recognition and uses the decision fusion method [33] to solve the fusion problem of two different modalities. The purpose of the decision fusion is to deal with the categories generated by each model and use specific criteria for redifferentiation. In the realization of this article, both facial expression recognition and speech emotion recognition use the Softmax function for classification. Their outputs are defined as

(12) $$\begin{array}{c} S^{\text{face}}=\left\{S_{1}^{\text{face}},S_{2}^{\text{face}},S_{3}^{\text{face}},\cdots ,S_{k}^{\text{face}}\right\}, \end{array}$$

(13) $$\begin{array}{c} S^{\text{speech}}=\left\{S_{1}^{\text{speech}},S_{2}^{\text{speech}},S_{3}^{\text{speech}},\cdots ,S_{k}^{\text{speech}}\right\}, \end{array}$$

where *k* is the number of emotional categories, and the weighted decision fusion calculation is

(14) $$\begin{array}{c} S=w_{0}S^{\text{face}}+w_{1}S^{\text{speech}},\;w_{0}+w_{1}=1. \end{array}$$

In the formula, *w*_0_ and *w*_1_, respectively, represent the weights assigned by the two modes.

## 4. Experimental Scheme

In order to verify the feasibility and practicability of the method mentioned above, the experimental simulation robot hardware environment is a Lenovo ThinkPad E14, AMD Ryzen 7 4700U 8-core processor, 16 GB RAM, and integrated graphics. The software environment is operating system Chinese Windows 10 and English version software Microsoft Visual Studio 2012.

This paper uses the Caffe deep learning framework to implement model training and testing on the MAHNOB-HCI data set. The data of 35 experimental participants in the MAHNOB-HCI data set is divided into training set A, validation set A1, and test set B at a ratio of 5 : 1 : 1. In the process of data preprocessing, the face video of the data set is downsampled to 8 fps. At the same time, the face image in the video is detected and cropped, and the image size is rescaled to 300 × 300. In the training process, this paper uses the Adam method [24] to update the parameters. The sample set used for each update is obtained by extracting a minibatch = 12 samples from the training set A through the experience playback mechanism. In order to prevent the model from overfitting, the value of the dropout is set to 0.5. Set the value of the maximum time step Nmax to 30. In addition, all fine-tuned VGG-16 networks used in this article have fixed parameters and are only used to extract features. In the experiment, rotation, flip, color distortion, and image transformation are used to expand the data. The whole data set was initially trained for 100 cycles with a batch size of 50. The initial learning rate of the model is 0.015, which is set to 0.001 after 10000 iterations. Set the weight decay and momentum to 0.00015 and 0.87, respectively. It is worth noting that the deep emotion recognition model is trained using a stochastic gradient descent scheme.

### 4.1. Sentiment Recognition Model Optimization and Analysis

#### 4.1.1. The Effect of LSTM Stacking Layers on System Recognition Rate

In order to explore whether the number of LSTM layers will improve the experimental results accordingly, this paper is based on the baseline model to conduct comparative experiments under different layers of LSTM.

Figure 6 shows the effect of LSTMs with different layers on the recognition rate of the system. Experimental data shows that, compared with a single-layer network, a multilayer LSTM has a better recognition effect and can better extract abstract features in a sequence. When *L* = 5, the recognition effect on the selected data set is the best, and the recognition rate can reach 0.89. When *L* > 5, the displayed effect gradually decreases. Therefore, the number of LSTM layers selected in this paper is 5.

#### 4.1.2. The Effect of Hierarchical Attention Mechanism on System Recognition Rate

After introducing the attention mechanism, different levels can be selectively paid attention to at each time step. In order to study whether the attention mechanism has a certain influence on the improvement of the network, this paper designs a corresponding comparative experiment.

As shown in Table 3, the introduction of the attention mechanism has improved the recognition effect of the model. After introducing the attention mechanism, the proposed model can achieve a high recognition accuracy of 0.89, which can increase the accuracy of 8.51% compared with the traditional LSTM model. In terms of the running time of the identification method, the proposed method can effectively be shortened by about 20 s compared with the traditional method. The attention mechanism is used to assign different proportions to each layer in the stacked LSTM, which is conducive to the network to filter out more useful information and improve the level of expression of the model and is more conducive to the extraction of image abstract features. Experimental results show that the introduction of the attention mechanism can improve the recognition effect.

#### 4.1.3. The Impact of Penalty Items on System Recognition Rate

In the attention mechanism, the weight coefficient of attention is used to improve the recognition effect. Among them, the addition of penalty terms *α*_*ti*_ and *β*_*ti*_ can be used to update the weight coefficient, and the recognition models obtained by different weight coefficients are different. By introducing variance, the difference between different weight coefficients is obtained, and then, the back propagation algorithm is used to maximize the variance.

In order to analyze the sensitivity of different penalty terms *α*_*ti*_ and *β*_*ti*_ in the proposed model to optimize the model parameters, the MAHNOB-HCI data set recognition task was verified experimentally.

The optimal values of model parameters are analyzed in the self-collected data set, as shown in Figure 7. In the first experiment (a), *α*_*ti*_ was fixed at 0.001 according to the setting of multiple experiments, and *β*_*ti*_ was changed in [0.1, 0.2, 0.3, 0.4, 0.5, 0.6, 0.7, 0.8, 0.9, and 1.0] to learn different models. It can be observed that the accuracy of the model generally increases first, reaches the maximum value at 0.7, and then decreases. The results show that when *α*_*ti*_ is set to 0.7, the network model has no effect on parameter selection.

Experiment (b) fixed the value of *α*_*ti*_ to 0.7 and changed *β*_*ti*_ in the set [0, 0.0001, 0.0005, 0.001, 0.005, 0.01, 0.05, and 0.1] for comparison experiments. The results show that the recognition performance is very sensitive to the value of the parameter *β*_*ti*_, and *β*_*ti*_ = 0.005 guarantees the excellent recognition performance of deep learning features.

### 4.2. MAHNOB-HCI Data Set Identification Analysis

Based on the above determination of the model structure and related parameters, this paper uses the MAHNOB-HCI data set to perform expression testing on the final fusion network. The confusion matrix of the final identification result of the test set is shown in Figure 8. Each row represents the category to which the video really belongs, and each column represents the category given by the fusion network.

It can be seen from Figure 8 that the expression-EEG interaction model proposed in this paper performs very well in identifying “happy” and “surprise” samples, and the recognition accuracy can reach 0.95 and 0.92, respectively. In addition, it can be noticed that the fusion network has a low ability to recognize expressions of “disgust,” but the recognition accuracy rate also reaches 0.79. As can be seen from the above figure, most “disgust” samples are mistaken for “anger,” “happy,” and “sadness,” while most “sadness” samples are classified as similar emotions, such as “anger,” “disgust,” and “fear.”

### 4.3. Comparison of Facial Expression Recognition Classification Algorithms in MAHNOB-HCI Data Set

The MAHNOB-HCI data set contains expression signals and EEG signals. In order to ensure that the signal characteristics in each modal can better reflect the emotional information of the modal, the characteristics of the two signals are, respectively, fused to obtain the fusion characteristics representing each modal. The MMDDN method in reference [24], the MERML method in reference [25], and the method proposed in this paper have different methods for fusing multimodal features. The two method models are classified and identified under the MAHNOB-HCI data set, and the results are shown in Figure 9.

As shown in Figure 9, the proposed method has a higher accuracy in the classification and recognition of various emotions than the comparison method. The recognition accuracy rates of “anger,” “disgust,” “fear,” “happy,” “sadness,” and “surprise” were 0.82, 0.79, 0.83, 0.95, 0.82, and 0.92, respectively.

Based on the above analysis, compared with other methods, the multimodal fusion feature obtained by separately fusing each modal feature in this paper has better performance in emotion recognition. It shows that with the reduction of the cost of multimodal feature selection, the classification performance of each emotion is also improved to a certain extent.

## 5. Conclusion

Multimodal emotion recognition is an important and challenging research problem in human-computer interaction. Facing the accuracy and real-time requirements of emotion recognition, this paper proposes a deep learning-based expression-EEG bimodal fusion emotion recognition method. This method is based on the improved VGG-FACE network model to realize the rapid extraction of facial expression features and shorten the training and learning time of the network model. The wavelet soft threshold algorithm is used to remove artifacts from EEG signals to extract high-quality EEG signal features. Then, the signal features extracted in the expression-brain electrical bimodal state are based on the long and short-term memory network model and the decision fusion method to realize the final bimodal fusion emotion classification and identification research. In terms of the running time of the identification method, the proposed method can effectively be shortened by about 20 s compared with the traditional method. The attention mechanism is used to assign different proportions to each layer in the stacked LSTM, which is conducive to the network to filter out more useful information and improve the level of expression of the model and is more conducive to the extraction of image abstract features. Experimental results show that the introduction of the attention mechanism can improve the recognition effect.

Analysis of the experimental results shows that the proposed method can reduce the model emotion recognition time by about 20 s compared with the traditional method, and the accuracy of the six typical emotion recognition can be maintained above 0.79. The focus of future research will be to explore the platformization of the proposed method and strive to realize the commercialization of the proposed method.

## Figures and Tables

**Figure 1:** Recognition system framework based on VGG-LSTM network model.

**Figure 2:** Schematic diagram of attention mechanism.

**Figure 3:** Schematic diagram of hybrid model.

**Figure 4:** Schematic diagram of piecewise linear transformation.

**Figure 5:** Schematic diagram of comparison before and after EEG signal processing.

**Figure 6:** The recognition accuracy of LSTM under different layers.

**Figure 7:** Model parameter sensitivity analysis.

**Figure 8:** Schematic diagram of the confusion matrix of the MAHNOB-HCI data set.

**Figure 9:** Emotion recognition accuracy rate under different methods.

**Table 1:** Experimental simulation results of fine tuning of each model.

Network model	Pretraining data set	FER 2013 test set results (%)	SFEW test set results
Baseline DCNN	Null	56.21	54.35
GoogLeNet	ImageNet	61.23	59.21
CaffeNet	ImageNet	67.41	56.22
Residual network	ImageNet	72.34	68.34
VGG	ImageNet	76.21	71.23
VGG-FACE	Faces	89.21	78.24

**Table 2:** Correspondence of electrode code.

Symbol	Name
Fp	Front pole
F	Frontal
C	Central
P	Parietal
O	Occipital
T	Temporal

**Table 3:** Identification accuracy rate under different processing conditions.

Treatment conditions	5-layer LSTM	
	Recognition accuracy	Running time (s)
Ordinary	0.82	121.34
Add attention mechanism	0.89	102.31

## Data Availability

The data included in this paper are available without any restriction.
